# Rapid Policy Network Mapping: A New Method for Understanding Governance Structures for Implementation of Marine Environmental Policy

**DOI:** 10.1371/journal.pone.0026149

**Published:** 2011-10-14

**Authors:** John Michael Bainbridge, Tavis Potts, Tim Gerard O'Higgins

**Affiliations:** Centre for Coastal and Oceans Governance, Scottish Association for Marine Science, Oban, Argyll, Scotland; Institute of Marine Research, Norway

## Abstract

Understanding the relationships and dependencies in the development and implementation of environmental policy is essential to the effective management of the marine environment. A new method of policy network analysis called ‘*Rapid Policy Network Mapping*’ was developed that delivers an insight for both technical and non-technical users into the lifecycle, relationships and dependencies of policy development. The method was applied to the Marine Strategy Framework Directive and the Water Framework Directive in the UK. These case studies highlight the environmental policy challenges to protect the UK's marine coastal environment and they identify differences in the styles of policy implementation between the devolved authorities of the UK. Rapid Policy Network Mapping provides an opportunity to create a collaborative policy data environment with a relatively small investment. As a tool for civil society it should assist in their ability to understand and influence policy making and implementation.

## Introduction

The necessity to account for environmental benefits generated by ecosystems has long been recognised [1] and with continuing environmental decline [2] this has led to: ever increasing efforts to include ecosystem services in the policy making process; a move away from a sectoral approach; and the integration of social and ecological concerns in the management of the environment. Environmental management which incorporates such considerations is known as the Ecosystem-based Management Approach (EA) and is rapidly moving from theory to practice. Tallis et al (2010) [3] point to the need for multi-sectoral engagement, valuation of ecosystem services and recognition of the tight coupling between human and ecological well-being for the effective delivery of EA. Crowder and Norse (2008) [4] support this view and propose a place-based ecosystem management approach where governance systems provide an incentive for stakeholders to be aligned. The need for transparent decision making which is inclusive of stakeholders at all stages and enjoys high levels of cooperation and coordination is critical to meaningful development and implementation of EA [3].

While the theoretical ecological and economic basis for the EA continues to grow at pace, implementation of the EA requires that the existing policy making and delivering institutions must be able to accommodate and adapt to a new multi-sectoral approach. Understanding how existing institutional structures function is an important first step towards this adaptation. It will require a move away from the traditional linear and ‘*command and control*’ approaches to delivering science into policy, demanding instead a more dynamic understanding of engaged and relevant institutions and the policy development process [5]. The Scottish Government define key stakeholders as including ‘*individuals or bodies with expertise/interest in a specific policy, or cross-cutting policies, whose contribution should be sought by officials to ensure policies and services meet the diverse needs, priorities and expectations of the people of Scotland.’* [6]. In their white paper preceding the UK Marine Bill the UK Government stated in 2007 that: ‘*Marine Planning will be an inclusive process for all interested stakeholders*’ [7]. Potential impacts on stakeholders from changes in the management of the marine environment range from loss of livelihood and the removal of existing access rights, to improvements in water quality and economic opportunity. Implementation of an EA in the Europe's regional seas poses its own unique set of challenges because the Union is made up of independent nations with their own languages, cultures, histories, institutional structures and economic objectives as well as diverse attitudes and perspectives toward the marine environment – a complex recipe to feed into coastal and marine planning.

The EU vision for future management of its seas is set out in the “*Blue Book*”, the Integrated Maritime Strategy of the EU [8]. The EU Integrated Maritime Policy (IMP) calls for “*integration of maritime governance*” to ensure stakeholder engagement, coherent agendas, removal of sectoral policy thinking and creation of cross-sectoral management structures [9]. Implementation of an EA, through the Marine Strategy Framework Directive (MSFD) [10] forms the environmental pillar of the IMP. The MSFD is one of the largest and most ambitious attempts at implementing the EA on an international scale and mandates its implementation in each of Europe's regional seas (Baltic, Black, Mediterranean and North East Atlantic) and for all EU member states. Despite a common obligation to implement the MSFD, there are numerous potential conflicting objectives both within and between nations. The Directive obliges each member state to achieve Good Environmental Status (GEnS) within their Exclusive Economic Zone by 2020 based on eleven environmental descriptors covering various aspects of environmental health as well as addressing anthropogenic concerns [11]. Targets for each of these descriptors will be set in 2012 and a program of measures to achieve these targets must be in place in each member state by 2016. The legal status and tight time-lines associated with the directive place an immense burden on scientists and on decision makers to put in practice a multidisciplinary approach, and will test the abilities of existing institutions to collaborate on delivering multi-sectoral objectives.

The MSFD assumes cooperation on a regional seas basis between member states as well as non-EU countries and promotes the use of existing institutional structures such as the regional seas commissions (HELCOM, OSPAR and the Black Sea Commission). At a state level many of the governance structures currently in place to manage Europe's coastal seas have been strongly influenced by the EU Water Framework Directive (WFD) [12] which deals with the ecological status of rivers and lakes as well as estuarine and coastal waters. The MSFD expands on the geographical scale and environmental scope of the WFD and contains a shift in focus toward integration of sectoral interests with the requirement to provide protection to *‘...aspects of the environmental status of the marine environment... not already addressed through Directive 2000/60/EC’* (the WFD) [13]. Whilst the transposition and implementation of the WFD has benefitted from the experience and evolved processes and policies of land planning across Europe [14], marine spatial planning is a relatively recent initiative with a limited legacy of successful implementation. Land planning benefits from private land tenure rights and the decisions made by local planning authorities typically consider most social, economic and environmental aspects of any proposal, including community opinion [15]. Key differences between marine and land planning include the three-dimensional nature of the sea; issues of ownership; usage rights; multiple-use; and the scale and remoteness of the marine environment [16]. Land-use planners might be expected to be involved with marine planning to the extent for which they are legally responsible and this is reflected in proposals for the English marine regions which include four non-coastal areas out of a total of 10 regions [17]. The geographical and political scale encompassed by the MSFD is significantly different from the WFD and implementation must accommodate the needs and wants of a greater number and dispersed set of stakeholders.

The economic and environmental research challenges involved in delivering GEnS are significant and will require extensive stakeholder consultation, engagement and participation [18] as well as necessitating a high level of change and development of institutional structures and policy networks. The future environmental status of European seas (and the success or failure of the directive) is therefore highly dependent on governance structures and policy networks. Attaining EA through the MSFD requires a holistic approach recognising the interconnections between the natural environment and human activities and institutions. It is conceivable that the imposed pressure to establish measureable GEnS parameters by scientists and politicians will shortcut meaningful stakeholder engagement given the deadlines in place for implementation. An aim of this article is to show the relational networks between policy actors and policy instruments and to shed light on how the governance framework could better facilitate a meaningful approach to engaging EA to delivery of the MSFD.

A policy network may be defined as the congregation of interdependent governmental and non-governmental actors who share interests in public policy development and are ‘*institutionally either formally or informally linked’* [19] where linkages exist between actors and represent a flow of resources [20]. Modern democratic policy making is experiencing a trend towards governance, driven by the need to integrate multi-sectoral concerns, and an increasingly diverse range of governmental, private and non-governmental actors are becoming actively engaged in the policy development process [21]. Friedman (2006) [22] proposes that *‘...public policies are determined by a combination of legislative actions and (the) actions of implementing organisations...*’ which often include market forces and non-governmental organisations (NGO's) - the so called ‘*Civil Society’* [23]. Policy networks are formed as an integral component of the process of government [24] and the ability to achieve social, economic and ecological targets in the marine zone is dependent on the efficiency of governance and the structure and function of relevant policy networks. Where there exists a network of policy actors, then a related network of policy instruments may also be found. Links between actors are made on the basis of a number of factors including political opportunity, institutional roles, preference similarity, reputation, transaction costs, influence and social trust [25]. The motivation and engagement of individual policy actors is driven by their perceptions and assumptions [26]. Policy implementation is subject to discretionary decision making which may result from a constraint on available resources and/or interpretation by individuals and organisations at the delivery level as described by Lipsky (1980) [27]. With many government policies competing with other organisations for resources and priorities, this can rapidly lead to de-prioritisation, the loss of (central) control and apparent policy failure [28].

Policy Network Analysis is a form of Social Network Analysis (SNA) that can provide an insight into the balance and patterns of responsibility, accountability, authority, resources, relationships and power in a policy process [29]. SNA typically considers a defined population within a prescribed policy ‘*boundary*’ and provides a robust analytical platform to better understand the dynamics and attributes within the defined community [30], [31]. In SNA, actors' attributes and relationships may be presented in graphical format using ‘*nodes*’ and ‘*ties*’, where a node represents an actor and the ties (links between nodes) portray the strength, direction and intimacy with other actors in the network [32]. SNA can provide insight into the strength, concordance and resource flows between actors, as well as providing information on actor importance, centrality, influence, contagion and dependency [33]. Actor densities provide an understanding of resource exchange within the network as well as insight into actor cohesion on particular issues and interests [34].

Policy network analysis has evolved to become a specialist area of study with established protocols, software and techniques available to facilitate the collection, manipulation and interpretation of data, often requiring dedicated resources and expertise. Such methods are presently limited in supporting day to day decision making in marine planning and in the communication of policy information to a non-technical audience. Whilst this paper acknowledges SNA as a robust analytical approach, it identifies a niche in terms of delivering a simple, rapid and pragmatic alternative to capture and provide insight into institutional dynamics and policy information. We present a new method to examine policy networks, called Rapid Policy Network Mapping (RPNM) and have applied it to the EU's Water Framework Directive and Marine Strategy Framework Directive, specifically in England and Scotland. The UK policy environment provides an excellent opportunity for policy network analysis due to the devolved administrative structure whereby limited autonomy exists between regional governments. The RPNM method was developed to allow non-specialists to quickly establish an understanding of the policy context within which they are working and to create a useful ‘working tool’. It provides a baseline assessment of a policy process in an easily understood and accessible format without the need for dedicated knowledge or skills. The RPNM approach aims to be information rich, detailing the content of policy instruments, their position in the policy making process, while specifying the role of actors in implementing policy decisions. The method results in an interactive resource which can be generated relatively quickly and made available to all stakeholders to provide a platform to support policy negotiations; further research; gap analysis; data storage; teaching; and communication. It allows stakeholders to visualise the social-economic, regulatory and legal structures inherent in management planning and to identify power relations between actors, and collaborate on solutions.

## Methods

The RPNM method was used to map and analyse the network of relations between policy actors and between policy instruments in the context of implementation of the MSFD and WFD in the UK. Based on the assumption that a significant majority of actors in a policy network are known to each other, the approach begins by analysing the documents of a single organisation, and follows a chain of references from this point. This method adopts an ‘*ego-centric approach*’, where an ‘ego’ is a policy actor or instrument linked to other relevant policy actors and instruments in a policy community and where the ‘*centrality*’ of the instrument or actor is a function of its importance within that network. This approach is traditionally used to sample large populations based on the assumption that actors are typically known to each other and has been used to explore issues including heritable traits, drug abuse and behaviours [35].

Policy instruments, reports, planning documents, organisation websites and policy statements pertaining to the two European Directives were analysed and the relationships and dependencies of policy actors and instruments were simultaneously identified, categorised and recorded. The study began with a single policy actor and based on referrals from this source, information on linked, related or dependent policy actors and instruments was gathered, but only if referenced in the context of the policy under investigation, i.e. the WFD or MSFD. Each of these referenced actors and instruments was then used as a new starting point and the process repeated. When referrals ceased to reveal new actors or instruments related to the relevant directive the process was terminated. This peer nominated approach is known as the “*Snowball Technique*” [35], [36].

Policy actor and instrument data was collated in Microsoft Excel (available on request). It was necessary to develop mapping templates for the actor and instrument policy communities to ensure consistency of reporting. A series of visual templates were created using CmapTools software (http://cmap.ihmc.us/), a “*knowledge modelling kit*”, developed by the Institute for Human and Machine Cognition [37]. The gridded templates provided a matrix for collating policy actors and instruments as a function of categories, domains and definitions described below, linked to the policy process flow. Relationships between actors or instruments were reported using ‘ties’. The templates provided a means to generate network maps allowing process flows and relationships to be visualised. The use of CMapTools facilitates unrestricted user access; public sharing, and synchronous updating and linking to other relevant CMaps.

In the actor template (figure 1) the columns delimit international to local policy domains with all actors linked to the policy process flow (described from left to right in the second row). Policy ‘influencers’ were reported above the process flow and three other categories of policy actors were reported underneath (described below, see table 1). No vertical hierarchical structure in the templates, for either the actor or instrument categories, is assumed. The instrument template (figure 2) was designed similarly with vertical columns to display policy domains and the policy instrument categories (described below, see table 2) were captured in rows so that a comparison of the actor and instrument policy maps was possible. The policy instruments for the UK and devolved authorities were separated into Acts, Regulations and Orders & Guidance to reflect the process of policy implementation in the UK.

**Figure 1:** Example of the policy actor template. In the actor template the policy process flow is from left to right and this is mirrored by the policy domains of actors from international on the left through to local actors on the right. The rows aggregate actors on the basis of the categories described in table 1.

**Figure 2:** Example of the policy instrument template. In the instrument template the policy process flows from left to right as international objectives are interpreted, transposed and implemented across the policy domains described in the columns. The six categories of policy instruments are aggregated in rows. These instrument categories are: General-water/marine specific; General-linked to directive; Environmental and biota related; fisheries; pollution-source/sink and planning.

**Table 1:** Categories of policy actors.

Actor	Definition
Influencer:	An organisation, entity or individual which is legally, morally or practically required, invited or obliged to be involved in the official policy development process. This does not include organisations, entities or individuals responding to a public consultation process, or similar, if they are not legally, morally or practically required, invited or obliged to be engaged in the official policy development process. It is assumed that Influencers can affect the outcome of the policy process using legitimate means based on their opinions and views.
Owner/Decision Maker:	An organisation, entity or individual which has the authority to make a *decision* which can affect the policy outcome as concerns intellectual or practical components or which *owns* all, or component parts, of the policy development process within a specified boundary. The majority of these actors are responsible and accountable for the successful delivery of intellectual and/or practical objectives which may include reporting, data, legislation etc. Decisions may be made by Owner/Decision Maker's following consultation and/or negotiation however it is assumed they have the ultimate authority to decide outcomes.
Influencer/Deliverer:	An organisation, entity or individual which is legally, morally or practically required, invited or obliged to be involved in the official policy development process. They can affect the outcome of the policy process using legitimate channels based on their opinions and views and are also engaged in delivering an action, process, or report which facilitates the interpretation, transposition and/or implementation of the policy.
Deliverer:	An organisation, entity or individual which is legally, morally or practically required, invited or obliged to be involved in the official policy development process. They can affect the outcome of the policy process based on their delivery of actions, processes or reporting which facilitate the interpretation, transposition and/or implementation of the policy. They cannot, in principle, affect the outcome of the policy process based on their opinions and views.

In order to simplify the mapping output the policy actors were categorised in terms of their responsibility to deliver an output; to influence the policy development; or to make decisions as ‘owners’ of a component of the policy process as defined here.

**Table 2:** Definitions of policy actor and policy instrument domains.

Actor Domains:	Instrument Domains:
International	International
European	European
United Kingdom	UK, all authorities: Acts
United Kingdom component (national) authorities: Scotland, Northern Ireland, Wales and England.	UK, all authorities: Regulations
Sub-National	UK, all authorities: Orders and Guidance

Policy actors and instruments were aggregated by policy domain using the definitions described here to allow comparison.

Actors were aggregated in categories to reflect their responsibility to deliver an output; to influence policy development; or to make decisions as ‘owners’ of a component of the policy process (table 1). Relationships between actors were not reported unless explicitly stated in a referred source. Policy actors were grouped according to their “policy domain” defined by international, national, regional or local scales. Where a number of actors from different domains were related or dependent via an advisory or reporting group they were linked to an actor group node highlighted in a primary colour, thus allowing communities of policy actors from different policy domains to be recognised as a coherent group (see case study actor map for WFD Scotland on Cmap servers). All advisory/reporting group nodes were only linked to the policy process where that group had an impact within the policy development process to avoid visual over-complication.

Policy instruments were aggregated according to the following six categories; ***General-water/marine specific***; ***General-linked to Directive***; ***Environmental and Biota related***; ***Fisheries***; ***Pollution-source/sink*** and ***Planning*** and by policy domain, linked to the policy lifecycle, as defined by the following phases: creation, interpretation, transposition and implementation (table 2).

In addition, organisations which had engaged in public consultations, but were not an active actor in the policy community, were recorded in the Excel spread sheets for completeness and to support future research (available on request). The model was applied to three European policy development processes: the MSFD for the UK, the WFD for the Anglian River Basin Management District in England and the Scotland River Basin Management District (for Scotland). The case studies used the following policy actor ‘seed ego's’: the Scottish Government; the UK Department for Environment Food and Rural Affairs (Defra) and the UK Environment Agency. Core documents on the respective websites of these three policy actors were used to originate the policy instrument mapping information. The data presented in this paper reflects policy landscapes of the MSFD and WFD up to September 2010.

## Results

The policy mapping templates provide a flexible basis for application of RPNM to policy problems. In total six Rapid Policy Network Maps were generated which may be examined in detail online using CMAP software and CMAP online servers or by visiting the KnowSeas Project web site and are listed below.

1. Marine Strategy Framework Directive; policy actor network map.
2. Marine Strategy Framework Directive; policy instrument network map.
3. Water Framework Directive; policy actor network map for the Anglian River Basin District.
4. Water Framework Directive; policy instrument network map for the Anglian River Basin District.
5. Water Framework Directive; policy actor network map for the Scotland River Basin District.
6. Water Framework Directive; policy instrument network map for the Scotland River Basin District.

In order to access the online CMAPS, download the CmapTools software from http://cmap.ihmc.us/ (accessed 2011 September 22) and open the file RPNM which is found in the ‘IHMC Public Cmaps’ in ‘Shared Cmaps in Places’. Alternatively, you can view the Cmaps for these Directives as PDF documents on the KnowSeas web site here: http://www.knowseas.com/links-and-data/rapid-policy-network-mappping (accessed 2011 September 22).

Only the Scotland WFD policy maps show policy domains to a local level (Argyll) to capture policy actors represented in Area Advisory Groups and a direct comparison between England and Scotland processes should be made excluding this domain.

The MSFD actor map (Map 1) is an attempt to map the key policy actors and institutional architectures at a particular point in time, in this case from June to September 2010. The map charts the array of actors involved in the policy development of the MSFD at the UK policy scale who were cited using the snowball method and with the caveat that this did not capture all actors engaged in marine policy in the UK. This period was early in the UK development process and during the transposition of the Marine Strategy Regulations 2010 [38] that established the overarching policy process at the UK scale. The MSFD actor map shows a more barren actor landscape than the WFD (see maps 3 and 5) which has had a longer timeframe for policy development and application.

The MSFD actor map tells different stories about the UK policy actor landscape. In total, 80 different actors from the international to regional scale are involved in influencing or delivering policy on the MSFD (Table 3). At the EU scale, these are clustered around influencers and owner/decision-makers relevant to marine policy and involved in the broader issues of regulation, resourcing and coordination. For example, OSPAR is critical in providing potential coordination in the NE Atlantic to reach GEnS and the European Commission provides policy direction and support to all EU states, whilst ICES is a provider of scientific advice increasingly aligned to the ecosystem approach. At the UK scale the number of actors increases with transposition, with 59 actors across UK and regional scales and the balance occurring at the national and devolved scale in this assessment (in comparison to the WFD actor map with more emphasis on regional delivery). The map shows that while a number of actors influence policy, or deliver policy functions, the UK Government is the primary decision maker (and is ultimately responsible for successful delivery of the MSFD). The UK Government is advised by a number of key national scientific bodies such as the Marine Assessment and Reporting Group, the Marine Science Coordination Committee, and the Marine Climate Change Impacts Partnership who influence policy direction and implementation and are supported by a number of scientific delivery agencies such as Natural Environment Research Council (NERC) and the Marine Environment Data and Information Network (MEDIN).

**Table 3:** Summary results of policy actors for the three case studies.

		Policy Domain/Scale				
Policy Actor status	Directive	International	EU	UK	England, Wales, Scotland, or Northern Ireland	Local/sub-national
**Influencer**	WFD Scotland	1	13	11	30	10
	WFD Anglia	0	15	11	10	1
	MSFD UK	5	4	7	4	3
**Owner/Decision maker**	WFD Scotland	2	4	5	6	1
	WFD Anglia	1	3	7	3	4
	MSFD UK	6	4	6	5	2
**Influencer/Deliverer**	WFD Scotland	0	3	5	7	3
	WFD Anglia	0	2	7	8	12
	MSFD UK	0	0	1	5	2
**Deliverer**	WFD Scotland	0	0	0	9	0
	WFD Anglia	0	0	2	5	21
	MSFD UK	1	1	17	7	0

The respective numbers of policy actors are presented here by category and policy domain for each of the three case studies.

The instrument map for the MSFD (Map 2) highlights a complex policy landscape comprising 162 different instruments from the international scale to sub-national operational scales (Table 4). The instruments are relatively evenly spread across environmental categories with the most occurring in the water/marine domain, followed by biodiversity, pollution, general sustainability and fisheries. Planning instruments were the least represented but are important in terms of integration with the national and sub national planning framework and with further transposition into devolved contexts, the number of these instruments would be expected to increase. At the EU scale, 56 instruments dominate the policy landscape and directly or indirectly relate to the implementation of the directive, whereas at the UK scale in excess of 90 acts, regulations, orders and forms of guidance are identified that correspond to the delivery of the MSFD. The diversity of policy instruments highlight the complexity in administering a policy that cuts across the breadth of maritime sectors and draws upon a range of management tools from sectors as diverse as pollution control, biodiversity protection, fisheries and planning. The data points to a snowballing of effort as transposition from the international to sub-national scale increases the obligations, efforts and resources of member states and the complexity of achieving GEnS in marine and coastal environments. The instrument map highlights that marine policy integration and delivery will be an important aspect of the MSFD, requiring mechanisms to support horizontal and vertical integration which will be important determinants of success, particularly where there are limited resources. Instruments such as the Marine and Coastal Act 2009 [39] and Marine (Scotland) Act 2010 [40] have laid the foundations for marine planning and objective setting across multiple sectors and will likely mesh with MSFD objectives into planning efforts. The challenge to policy communities at the UK and devolved scales is to ensure a joined up approach within and between governments and the instrument map demonstrates the emerging complexity at an early stage of transposition at the UK scale.

**Table 4:** Summary results for the policy instruments for the three case studies.

		Policy Domain/Scale				
Policy Instrument Category	Directive	International	EU/European	UK: All Authorities - Acts	UK: All Authorities - Regulations	UK: All Authorities - Orders & Guidance
**General: Water/Marine Specific**	WFD Scotland	0	6	6	5	6
	WFD Anglia	0	6	7	4	2
	MSFD UK	1	17	6	11	6
**General: Linked to MSFD**	WFD Scotland	0	2	5	0	5
	WFD Anglia	0	2	5	0	0
	MSFD UK	1	8	11	0	7
**Environmental & Biota**	WFD Scotland	1	4	3	7	2
	WFD Anglia	1	6	7	0	2
	MSFD UK	6	6	3	15	1
**Fisheries**	WFD Scotland	0	5	3	2	5
	WFD Anglia	0	4	2	2	6
	MSFD UK	5	8	10	0	2
**Pollution, Source & Sink**	WFD Scotland	2	14	2	10	4
	WFD Anglia	2	14	2	15	10
	MSFD UK	3	14	5	7	1
**Planning**	WFD Scotland	0	4	9	14	20
	WFD Anglia	0	4	7	22	10
	MSFD UK	0	3	2	3	0

The respective numbers of policy instruments are presented here by category and policy domain for each of the three case studies.

## Discussion

The RPNM approach is an attempt to provide an additional mechanism to help facilitate the practice of institutional reform and aid delivery of an ecosystem approach to marine policy. As noted in Tallis *et al* 2010, [3] implementing the EA takes constant learning, adaptation and investment in the social and natural sciences. This study has mapped the policy context in two case study contexts (MSFD and WFD) and the novelty lies in creating a publicly accessible platform for collaboration on institutional awareness and reform. The maps provide an immediate sense of the size, complexity and scale of the policy actor and instrument communities involved in the three implementation processes in the UK. The translation of each directive to ‘local’ implementation appears to follow a hierarchical ‘*hand-over*’ of policy between domains (from left to right in the maps) which also reflects the lifecycle of the policy development process. This hand-over of policy processes at each scale inevitably involves political negotiation and institutional bargaining and is influenced by the legal capacity and influence of actors within each domain.

At a European level there are many more policy instruments in place for the MSFD than the WFD. The WFD has reached a relatively mature implementation stage whereas the MSFD is still at the transposition stage in the UK and does not appear, at the time of the study, to have driven the creation of significant numbers of new, dedicated UK level legislation, nor is there evidence of comparable numbers of actors yet engaged at UK devolved scales. In the WFD policy process 36 EU instruments catalysed 104 UK policy instruments (Table 4). If the implementation of the MSFD follows a similar trend to the WFD, then pro-rata the identified 56 EU instruments for the MSFD process will require the creation of up to 70 more UK policy instruments (this assumes that the two policies are of equal complexity and follow a similar pattern of implementation). A comparison of actor maps also highlights the difference in the life cycles of the two directives with the MSFD process showing significantly less actor engagement at a UK devolved level. This snapshot of the MSFD process in 2010 raises important implications for actor participation as implementation of the directive will likely need to engage with a higher number of stakeholders than the WFD. As the timetable for establishing objectives and targets get closer, there is a substantial need for user engagement in the process beyond consultation with a move to active partnership, particularly in light of the magnitude of challenges required to achieve GEnS. The assessment of the institutional and actor frameworks in 2010 suggests there is still considerable need for further reform. Many of the policy instruments and actors are common to the implementation of both directives e.g. the Habitat Directive and the UK Environment Agency, which should lead to greater efficiency in developing a programme of integrated policy delivery in the coastal zone. However, each Directive may be the responsibility of different groups and individuals within these actor organisations and any potential efficiency will be dependent on internal co-ordination and the quality of inter-actor relationships at an individual level [41].

The transposition of the MSFD lies at a critical juncture in the UK as the policy process is unwound in the devolved context and complexity, engagement and reform become real issues for authorities leading coastal and marine planning. As highlighted in the Convention of Biodiversity Malawi Principles for an Ecosystem Approach [42], management objectives are a matter of societal choice and management should be decentralised and multi-sectoral. Whilst the RPNM maps indicate that the MSFD transposition is poised to achieve this within the UK context the challenge is on how these processes will be operationalized. The enactment of the various UK marine acts offers scope for ecosystem based management reform and the evolution of regional marine planning, but only if regional plans and planning initiatives are adequately resourced, represented and given the authority to make decisions to manage the balance between conservation and appropriate use. Regional plans can provide the grounded coordination across maritime sectors and enable the management of policy complexity, however they will not work in a vacuum and there is a considerable opportunity for institutional cross learning to occur as shown by the actor and instrument maps in this study.

In recent years, Scotland, Wales and Northern Ireland have sought to exercise increased control over their respective policy jurisdictions and since devolution, both Wales and Scotland have adopted a partnership approach to policy implementation. They have done this by building close relationships between government and delivery organisations, typically with more flexible targets than in England. The Scottish Government continues to object to the perceived *‘coercive*’ transfer of UK objectives to the devolved authorities, particularly for reserved matters [43]. Following devolution, Scottish legislation is similar but not identical to that in England, Wales and Northern Ireland and so there is the potential for Scottish actor discretion in the transposition process, which has been reported in other European states, albeit that this is sometimes a result of legal architecture incompatibility [44]. England and Scotland WFD implementations have similar numbers of policy instruments related to their delivery despite the differences in legislation. The results for WFD implementation in England and Scotland show higher levels of cross-domain integration of policy actors in the Scottish implementation which was not apparent in the English process. This finding supports the opinion that the ‘*command and control*’ approach to governance found in England is not as prevalent in Scotland and this is reinforced by statements made by the UK Environment Agency in the Anglian River Basin documentation, specifically that: ‘...*the Environment Agency will need to identify specific environmental objectives for each water body and develop a river basin management plan which sets out what we and others need to do to achieve them.’* [45].

Successful implementation of the MSFD and international coordination through the regional seas conventions is an overarching UK responsibility. Delivery within the UK will be by the devolved authorities and at the time of map generation, this was an emerging policy issue and had not advanced in terms of policy development. The 2010 Regulations establish the UK architecture for MSFD implementation and hence many of the actors, consultations, and instruments were in an early stage of deployment. To complicate matters, negotiations between UK and devolved authorities over marine management and planning under the Marine and Coastal Access Act (2009) were occurring during this period, with a focus on the UK Marine Policy Statement that was launched in March 2011. The Marine Policy Statement enables a consistent approach to marine planning across UK waters and coordination amongst devolved governments (‘owner - decision makers’) and delivery agencies. The consultations on regional implementation are anticipated for December 2011 and whilst this increases the complexity of the engagement and implementation process, it also allows for decentralisation and democratisation of the decision making approach which is a hallmark of the ecosystem approach to management [3], [38]. The authors emphasise that new participatory and peer reviewed mapping exercises should be developed that capture emerging circumstances. MSFD implementation at the national and sub-national scale will draw upon an array of policy instruments and will require considerable coordination within and between government departments and agencies - the domain of horizontal governance. In addition, MSFD implementation will require mechanisms that deliver vertical governance efficiency ensuring that objectives are carried from the EU and transposed through national and sub-national scales and joined up into operational activities. Measures may take the form of inter-governmental agreements or joint monitoring programs that boost policy cooperation (for example the Marine Assessment and Reporting Group that are identified in the actor map). Parliamentary reviews and independent audits by civil society or commissions such as the Audit Commission in Scotland will add a level of transparency and act as a means of performance review.

## 

### Conclusions

The approach of the WFD has been to address components of the ecosystem separately whilst the MSFD demands that the whole of the ecosystem is considered based on the 11 descriptors of GEnS. Borja et al (2010) [46] point to these key differences between the WFD and the MSFD and describe them as a ‘*deconstructing structural approach’* and a ‘*holistic functional approach*’ respectively. If the MSFD is to be implemented using an ecosystem based approach and embrace the holistic functional approach it sets out to achieve, then this suggests that a high level of stakeholder engagement, in and across all policy domains, would be necessary from early in the policy transposition and implementation process and during the development of the GEnS indicators. Based on the results of this analysis, this is not the case as there is no evidence of significant inter-actor engagement in, and between, policy domains, or of the engagement of sufficient sub-national stakeholders in policy transposition, implementation, planning or development of GEnS descriptors. The MSFD was written into EU law in 2008 and the determination of environmental targets needs to be set down by EU members by July 2012. In the UK, whilst the scientific and political communities are establishing the standards and environmental targets for public consultation in 2012, initiating public consultation at this late stage does not satisfy the need for ‘*multi-sectoral engagement, valuation of ecosystem services and a tight coupling between human and ecological well-being’* [3]. An ecosystem-based approach would expect public consultation and active partnerships to have engaged with the process from the early transposition phase, as shown in figure 3.

**Figure 3:** Timeline for the Marine Strategy Framework Directive. The timeline of implementation is established for all EU member states within the MSFD. If an ecosystem-based approach had been adopted from when the directive passed in to law in 2008, then the proposed public consultation i.e. stakeholder engagement, would have been applied in 2008 instead of the current plan to commence this process in 2012. The dotted box and arrow reflects the move of public consultation to 2008.

This study highlights the lack of stakeholder engagement in the implementation of the MSFD at all the relevant (and necessary) scales. Whilst there is a trend to empower local authorities in the UK, none have yet been included in the process to define GEnS. Effective representation of multi-sectoral goals (a pre-requisite for the ecosystem approach) within the MSFD would be represented in the RPNM maps by an increased number of multi-sectoral actors from all policy domains linked to the left hand side of the policy maps. Future policies to implement EA might focus on setting goals and targets at the more local level, with a stakeholder led process propagating from local spatial scales upwards toward a unified European vision and legal formalisation.

The MSFD shares policy actors and instruments in common with the WFD and with many other relevant EU Directives. A comparison of these Directives using RPNM would provide guidance on which policy actors and stakeholders have a high likelihood of future engagement in the MSFD process. As marine planning and policy development attempts to respond to the threats to marine ecosystem health and sustainability, a plethora of research and implementation programmes have been initiated at the scale of catchment, coast and sea. An understanding of the policy context in which they operate is relevant to many of these programmes as it describes the role and structure of institutions, actors and instruments, and the relationships between them. Many stakeholders do not have the budget, resources or time to invest in an in-depth policy network analysis, nor do they require the level of information it might provide. It is hoped that RPNM will fulfil this role by providing a baseline assessment of a policy community in an easily understood and accessible format. This information can be used to chart policy and institutional strategies that recognise the complexity of social and political systems and the pathways to implementation and transparency and, in the case of the MSFD, provide guidance on stakeholder engagement.

The RPNM approach provides a platform for further research and the results provide a map of the governance system ‘as it is’ and are the basis for further discussions on ‘how it could be’. Using the collaborative features inherent in the conceptual modelling process in RPNM, stakeholders could discuss and identify means of improving democratic accountability, policy efficiency, and innovative institutional structures. The outputs of RPNM could be used by stakeholders and institutions to identify where political power resides within the policy system, and improve access to, and influence over decision making, by groups who have been left out of the process. While the RPNM process does not remove the hurdles from embedded power structures, it can make them clear and explicit, and improve negotiations about future models of implementation. The main benefits of RPNM are that it:

1. Captures the majority and most significant instruments and actors in the development of specific policies.
2. Aggregates actors and instruments by policy domain.
3. Provides a robust platform of data as a baseline for reference or further research or action e.g. multi-modal network analysis, inter-policy networks etc.
4. Provides a web based tool for dynamic collaboration.
5. Allows a comparison between policy actors and instruments, by policy domain.
6. Groups actors by their attributes, i.e. in terms of owner/decision maker, influencer or deliverer.
7. Groups policy instruments by their major focus.
8. Links instruments where there is a direct relationship.
9. Links actors by intra and inter-domain group and/or activity reflecting resource transfer between domains.

The method and tools used for this method of network mapping has a number of caveats:

1. The model does not claim to provide a fully comprehensive database and network map of all instruments and actors.
2. The maps do not capture actors or groups with a historical transitory engagement in the process, for example, a number of collaborative research and liaison groups were established and disbanded during the development of River Basin Management Plans and are not included.

A benefit of this web-based approach to policy network mapping is that it is easily replicated and the use of the Cmap platform means that the policy maps can be placed on Cmap servers for open collaboration to achieve a ‘peer reviewed’ real-time output. The possibility to add attachments (Directives, website links etc.) to each of the nodes means there is the potential to build a pro-active online data-warehouse and to build a catalogue of inter-related policy maps on a country by country basis. By saving maps at pre-determined intervals it would also be possible to observe the evolution of a policy and its associated actor and instrument communities over time.

Rapid Policy Network mapping provides a real opportunity to create a policy data environment based on a relatively small investment which would provide value to a large number of users. For policy makers it charts the pathways for policy implementation, collaboration and for reducing horizontal and vertical fragmentation. It may serve as a means of policy innovation when an understanding of the broader network reveals further options for delivery and efficiencies. With an increase of collaborative effort and data sharing there are options for policy learning between stakeholders, sectors, jurisdictions and nations over the implementation of the ecosystem approach in coastal and marine regions.
